# The Use of BP Neural Network Algorithm and Natural Language Processing in the Impact of Social Audit on Enterprise Innovation Ability

**DOI:** 10.1155/2022/7297769

**Published:** 2022-05-18

**Authors:** Jie Wang, Xiaomei Wang, Haili Wen

**Affiliations:** ^1^School of Economics and Management, Nanjing University of Science and Technology, Nanjing City 210094, China; ^2^School of Economics and Management, Chuzhou University, Chuzhou City 239000, China; ^3^Intellectual Property Institute, Nanjing University of Science and Technology, Nanjing City 210094, China

## Abstract

At present, there are still some problems in the document management of enterprise innovation projects, such as non-standard management, lagging update, chaotic content, insufficient information, and insufficient application. There is still a lack of effective methods to evaluate the financing ability of enterprises. To solve the above problems, high technology expertise (HNTE) is taken as the research objects. Firstly, the relationship between social audit and enterprise technological innovation is analyzed, and on this basis, combined with natural language processing (NLP), an extraction method of project document information is proposed. Secondly, the evaluation index system of enterprise financing ability is constructed based on Back Propagation Neural Network (BPNN), and the technology innovation audit system of HNTEs. Finally, combined with the actual content, the proposed document audit method is evaluated. The results show that: the average accuracy rate of the NLP-based innovation project document audit method is 91.36%, the average recall rate is 96.34%, and the average F statistical value is 95.34%. Among them, the recall rate and F statistical value are about 2.3% and 1.4% higher than manual processing, respectively. The recall rate and F value are obviously better than those of manual processing methods, and the processing time of single document based on NLP is only 87.5 s. The processing time is nearly 50 times lower than that of manual processing, which greatly improves the processing efficiency of document information. The corresponding test results of each index selected based on the evaluation of enterprise financing ability are all below 0.1, which meets the requirements of consistency. The evaluation results of BPNN model on enterprise financing ability are highly consistent with the target value, and the prediction error is controlled within 0.02, which can provide more accurate prediction results. This research obtains a more accurate prediction model of enterprise financing ability evaluation, which provides technical support for social auditing and the innovation and development of enterprise technology, and provides a feasible route for the development of BPNN in the financial field.

## 1. Introduction

In recent years, as the modern information technology develops fast, the market competition is further intensified, and higher requirements are put forward for the innovation level and innovation ability of enterprises. Comprehensively strengthening the leading role of scientific and technological innovation promotes the development of high technology expertise (HNTE) [1, 2]. However, at present, there are still some problems in the technology investment and management of HNTE regarding relevant innovation projects. There are still some problems in the document management of enterprise innovation projects, such as non-standard management, lagging update, chaotic content, insufficient information, insufficient application, and lack of effective methods to evaluate the financing ability of enterprises. Natural language processing (NLP) belongs to a type of artificial intelligence (AI) processing methods, which is originally originated from Turing test [3, 4]. The application of this technology can shorten the relationship between people and computers, so that computers can also read and write, which provides an effective idea for rapidly completing text data analysis and processing, key information extraction and so on. NLP can be further subdivided into Chinese word segmentation technology, named entity recognition, part of speech tagging, synonym analysis, and word vector analysis [5]. Obviously, NLP shows certain application potential in processing innovation project-related text and key information of HNTE. In recent years, deep learning (DL) has shown a rapid development momentum, and has excellent performance in the fields of feature extraction, image processing and so on. Among them, back propagation neural network (BPNN) is a typical representative of DL. The model belongs to feedforward neural network, which is a forward network formed by three layers or more structures. BPNN has excellent performance in prediction and other fields [6].

As for the application of NLP in text processing, Chatterjee et al. applied NLP and proposed a knowledge-based inter domain relationship extraction scheme. It was found that the reference parsing technology showed excellent performance in average accuracy and average recall rate, which were greater than 75% and 85%, respectively [7]. The continuous development of NLP technology has promoted great breakthroughs in the research of text processing algorithms. Text processing relies on the collaborative research of NLP and machine learning (ML) [8]. Abbaszade et al. obtained a machine translation model with a good translation effect by integrating neural network (NN) and NLP technology [9]. At present, many applications based on NLP have appeared on the market, such as voice assistants of smart phones, voice service systems of banks, etc. [10]. Regarding the application of BPNN in forecasting, Zhang, aiming at the aquaculture production and export, put forward a production prediction model based on optimized BPNN. The results showed that the root mean square error of the model was smaller than that of the traditional BPNN, and the learning efficiency was higher than that of the traditional BPNN. It showed excellent performance in processing abundant historical data, and could shorten the modeling time and obtain good prediction results [11]. Zhang et al. trained the BPNN by the differential evolution (DE) algorithm, and finally obtained a NN prediction model for the textile field, which provided technical support for the intelligent production of textile factories [12]. Zhang and Lou invented a NN model for industrial pattern classification based on BPNN and image processing technology, realizing automatic pattern recognition of industrial machines [13]. Based on the above results, it is found that NLP has been applied in text processing, and BPNN has shown good performance and application potential in the field of prediction.

However, there is little research on the application of NLP and BPNN in social audit, text processing of enterprise innovation project, and enterprise financing ability evaluation. Therefore, firstly, the study proposes an innovation project file audit method based on NLP to strengthen the document management of enterprise innovation projects and improve work efficiency. Secondly, an enterprise financing capability evaluation method based on AHP and BPNN is proposed to provide objective and accurate evaluation results of enterprise financing capability. Finally, it constructs the technological innovation audit system of HNTEs, and defines the audit theme, object, and overall audit process. The innovation lies in the combination of NLP and BPNN, which is applied in the innovation audit of HNTEs, providing significant technical support for promoting the development of enterprise technology innovation and optimizing social audit.

## 2. Method

### 2.1. Social Audit and Enterprise Technology Innovation

Chen et al. proposed that scientific and technological innovation is very important to promote economic growth and strategic security, and enterprises are the subject of scientific and technological innovation [14]. Social audit is a key component of the corporate governance and supervision system. The implementation of relevant audit procedures makes it possible to identify violations such as financial fraud. Thus, social audit plays a certain role in restricting a series of scientific and technological innovation activities of enterprises [15]. Among different types of enterprises, the so-called HNTEs specifically refer to the types of enterprises that are involved in industries within the specified high-tech fields and can continuously engage in corresponding research and development, and finally complete the transformation of relevant technological achievements. Such enterprises have independent intellectual property rights and belong to economic entities that concentrate technology and knowledge. For such enterprises, whether the relevant technological innovation activities can be held and implemented smoothly is affected by multiple factors, among which infrastructure, R&D funds, technical personnel, operation management, and production technology are the most important factors. These influencing factors are summed up, that is, the whole elements of enterprises' technological innovation activities. If classified by category, these elements can be divided into innovation input, capability, process, management, and output. Based on these innovation elements of corresponding enterprises, technological innovation audit is defined as audit subject relying on relevant methods. The laws and regulations and audit standards are taken as the basis, and audit opinions are proposed aiming at the audit of all elements of technological innovation in each stage and operation process. In this way, it is helpful to promote and improve the technological innovation system and mechanism of enterprises and further enhance the strength of technological innovation. HNTEs include many scientific and technological talents, which has high investment, high innovation, and high risk. Therefore, the social audit of technological innovation of such enterprises should emphasize the elements of technological innovation to achieve a more systematic and dynamic quantitative audit for the related technological innovation activities of enterprises.

Since the importance of technological innovation management in the development of enterprise innovation activities is considered, a method for extracting project document information based on NLP is proposed. For the development of HNTE-related innovation activities and social audit optimization, and based on BPNN, a growth value evaluation method based on the financing ability of HNTEs is proposed.

### 2.2. The Research Status of NLP

NLP is a technology that covers computer science, machine learning, and linguistics, which focuses on making people communicate with computers based on natural language. In terms of definition, NLP can be divided into two categories: natural language and processing. The whole processing process of NLP is to rely on computers to process the information of form, sound, and meaning. In the field of AI and linguistics, the realization of information communication between human and computer is a hot topic. In other words, one of the important purposes of NLP is to promote the interaction between computer and natural language understanding [16, 17]. The implementation of NLP mainly includes two stages: natural language understanding and generation. The former mainly represents the computer's understanding of the meaning of natural language text, while the latter realizes the expression of relevant definite intention based on the natural language text [18]. From the perspective of linguistics, NLP can be divided into phonetic, lexical, syntactic, semantic, and pragmatic analysis; from the angle of computer, NLP can be divided into four types: sequence tagging, relationship judgment, relationship generation, and classification [19, 20]. Shekhar et al. proposed a Hindi recognition technology by combining NLP with DL-based neural network model. The results showed that this technology had excellent performance in text language processing and accurate prediction [21]; Dreisbach et al. combined NLP and text mining to analyze the data extraction and processing of electronic medical records. The analysis of accuracy, recall, and F value indicated that the combination of NLP and data mining could be used to extract and analyze online symptom data [22].

For HNTEs, document management involving innovation projects is also very important. Compared with other types of document management, enterprise-related project document management has its own unique characteristics. The composition of project document management is diverse, and there is great demand for time efficiency and high requirement for security. However, there are still some problems in the management of project documents, such as not standardized management, lagging update, distorted content, insufficient information, and insufficient application. In view of the above problems, it is considered that the innovation project management in HNTEs should be mainly considered from the standardization, security, diversity, and timeliness. NLP has been widely used in AI text processing. In addition, the technology has good versatility, security specification, and strong timeliness, and can improve the ease of use of documents. Therefore, NLP is applicable in the document management of enterprise projects.

### 2.3. Evaluation of Enterprise Financing Ability Based on BPNN

The so-called neural network is a nonlinear system based on the simulation of biological reactions in human brain nerves, and then based on relevant sample data, it reasons concrete information, thus revealing the relationship between data and information. BPNN is an important method in the field of DL, and is also an important model in the neural network model [23]. BPNN not only has excellent prediction performance, but also has efficient solving ability. Wang et al. applied BPNN to predict the current of fuel cell and found that the proposed model had excellent performance [24]. Cui and Jing proposed a geotechnical parameter prediction model based on BPNN. Taking the engineering geological database as the platform and using MATLAB and other programming languages, they preliminarily studied and implemented the prediction model. The results showed that the generalization ability of the prediction model met the requirements [25]. These excellent performances are closely related to the composition and structure of BPNN. BPNN mainly consists of input layer, hidden layer, and output layer. The relevant information absorbed is promoted from the input layer of BPNN to the implicit layer, and then reaches the output layer under the action of information. At this time, if the corresponding output results meet the expectations, the current forward propagation can be completed. On the contrary, due to the existence of errors, the system will return the feedback results to the hidden layer to complete the reverse propagation. The repair purpose can be achieved by reducing the error, and the desired results can be obtained finally [26, 27]. In addition to the excellent performance in the prediction and solution level, BPNN also has good self-improvement, fault tolerance, and generalization ability. However, in the application process, BPNN has uncertainty, and high requirements for the selection of samples. If the network structure is uncertain, the output results will be affected to a certain extent because the weight proportion is not applicable.  Figure 1 shows the structure of BPNN. The typical three-tier structure of BPNN also endows it with the ability of nonlinear mapping, parallel operation, distributed storage, fault tolerance, self-adaptive ability, and comprehensive reasoning ability. Therefore, this method is applicable to the prediction and evaluation of enterprise's technological innovation capability. In view of this, BPNN is introduced into the evaluation of HNTEs' financing ability based on innovation investment.

As the financing ability of an enterprise is affected by multiple factors including innovation, profitability, management, growth, and security, these five factors are focused on, and more detailed indexes at this level are introduced.  Table 1 shows the realization of the specific financing ability index system.

### 2.4. Construction of Audit System for Technological Innovation of HNTEs

For HNTEs, the related technological innovation activities are professional, complex, and secretive. Therefore, the audit should focus on the combination from multiple levels. Based on different subjects, the audit can be divided into government audit, social audit, and internal audit. Government audit has authority, social audit has professionalism, and internal audit shows service introversion. Zhu and Li used information technology and internal control theory to make a detailed analysis on the operation status of China's HNTEs. The research suggested that HNTEs should strengthen the construction of internal control and financial accounting system [28]. In view of the innovation activities of HNTEs, the social audit is analyzed. The subject of the social audit is the accounting firm, which is a key component in the audit of enterprise technological innovation. The audit object is HNTEs with technology innovation. The technology innovation investment based on the financing ability is emphasized and the technology innovation management based on the innovation project management is taken as the main audit objects.  Figure 2 shows the audit content composition of total factor technological innovation of HNTEs.

### 2.5. Data Sample Selection and Processing

The effectiveness of the NLP-based audit method for innovation project documents of HNTEs is verified, and Table 2 shows the main clauses of the project document contract selected. Specifically, the effect of manual processing is compared with that based on NLP, and the evaluation indexes are precision (*P*) [29], recall rate (*R*) [30], and *F* statistical value [31].

Twenty HNTEs in Shenzhen Stock Exchange are taken as the research objects to analyze the innovation input and innovation management in total factor technological innovation. The idea of analytic hierarchy process (AHP) is applied, expert judgment method is used to judge the first-level composition index and the second-level composition index through constructing judgment matrix. Darko et al. proposed that the most prominent reason for using AHP was its small sample size, high consistency, and strong simplicity and availability of software operation [32]. The maximum eigenvalue and its eigenvector of the judgment matrix are calculated based on the algorithm, and the consistency test is made finally. The comprehensive score results of each enterprise are obtained through the weight of each index, and the financing ability of HNTEs based on innovation investment is judged. Based on the previous structural system, the 1–9 scale method is adopted, and the judgment matrix is constructed according to the affiliation between each level. Based on the expert judgment method, the judgment matrix for the pairwise comparison of different financing capacity indicators is shown in Tables 3 and 4, respectively.

Thirteen second-level indexes of 20 HNTEs are taken as the input of BPNN. The comprehensive score results are regarded as the output of BPNN, and the dimensionless data as the training samples to calculate the model, thus judging the effectiveness of BPNN in the evaluation of financing capacity of HNTEs. 1–9 are the importance comparison scales of the two indicators. The higher the importance, the higher the scale. The even scale indicates that the importance of the two indicators is between the two judgment scales.

## 3. Results and Discussion

### 3.1. Analysis of NLP-Based Innovation Project Document Audit

Based on the key clauses of innovation project document contract selected in Table 2, the precision (*P*), recall rate (*R*), and *F* value are used as evaluation indexes. The results of manual processing and NLP processing are shown in Figure 3. In Figure 3, *A*∼*N* represent the key clause numbers, and the specific content is the key clause number in Table 2, that is, *A* (Product name); *B* (Master slave relationship of product structure); *C* (Product operation form); *D* (Risk return characteristics); *E* (Investment strategy); *F* (Duration); *G* (Difference of subscription amount); *H* (Valuation base date); *I* (Minimum amount of individual initial subscription); *J* (Processing form of subscription interest); *K* (First differential); *L* (Pursue differential); *M* (Contractual securities broker); *N* (Redemption fee).

Figure 3 shows that after being processed by professional auditors, the average precision of the key clauses of the corresponding innovation project document contract is 95.29%, the average recall rate is 94.14%, and the average *F* is 94.05%. In contrast, the average precision of audit results corresponding to the key clauses of the NLP-based innovation project document is 91.36%, the average recall rate is 96.34%, and the average *F* is 95.34%. In terms of the overall processing time, the average time consumption of professional manual audit is 70 min, while that of single document based on NLP is only 87.5 s.

It is not difficult to find that, compared with manual audit, NLP-based audit method is significantly better in recall rate and F value, and its accuracy rate is only about 4% lower. However, regarding the overall processing time of innovation project documents, the difference between NLP and manual processing method is nearly 50 times. The further expansion of hardware resources can improve the processing efficiency of project documents. Obviously, NLP has outstanding performance in the processing time of project documents, and the application of this method has no restrictions on the project document template, which can realize batch processing, thus improving the processing efficiency of document information. Moreover, it is more comprehensive and systematic for searching key information of project documents, which can effectively avoid the situation that key information review is not in place, and can simultaneously improve the security, timeliness, and ease of use of important documents. NLP-based project document audit also provides ideas for optimizing and improving social audit.

### 3.2. Evaluation of Enterprise Financing Ability Based on Innovation Investment

According to the expert judgment matrix results in Tables 3 and 4, the normalized and eigenvector results corresponding to each primary index, and the weight distribution and consistency test results based on each secondary index are obtained (Figures 4(a) and 4(b)). The *I* on the abscissa in Figure 4(a) represents innovation; *P* means profit; *M* refers to management; *G* denotes growth; *E* expresses investment guarantee. In the legend of Figure 4(a), *I*_*s*_ indicates the normalized result of innovation index; *P*_*s*_ stands for the normalized result of profit index; *M*_*s*_ means the normalized result of management index; *G*_*s*_ denotes the normalized result of growth index; *E*_*s*_ shows the normalized result of investment guarantee index.

The normalized results of the five first-level indexes in Figure 4(a) are not very different. The eigenvector curve has little fluctuation, the eigenvectors of profit index and investment guarantee index are larger, the eigenvector of management index is second, and the eigenvector of innovation index and growth index is the smallest. In Figure 4(b), the change of the second-level index data reflects that the maximum value of the eigenvector corresponding to each primary index judgment matrix is 5.193, which appears in *G*2, which is the net profit growth index. The consistency test results of different second-level indexes manifest that the selected second-level indexes have satisfactory consistency, and the corresponding test index values are all less than 0.1.

Table 5 shows the weight distribution results of the corresponding first and second-level indexes.

Based on the comprehensive weight results of the above corresponding indexes, the comprehensive score results of the research company can be obtained after weighting these dimensionless data (Table 6).

The above scoring results suggest that the quantitative analysis of the financing capacity of HNTEs can be realized, and the strength of a certain enterprise's financing ability can be judged to make the corresponding analysis on the technological innovation investment of the enterprises explored. Technological innovation investment is a key link in the whole elements of enterprise technological innovation. Meanwhile, it is helpful for optimizing and improving social audit and related favorable policies. Based on the analysis of the financing ability of enterprises, for HNTEs, based on its own actual situation, further expanding R&D and ensuring continuous innovation can improve market competitiveness and financing capacity.

### 3.3. Evaluation of Enterprise Financing Ability Based on BPNN

Figure 5 shows the comprehensive evaluation results, network fitting errors, and network prediction errors based on BPNN obtained with the second-level index as the input and the comprehensive score as the output.

As Figure 5 shows, the black line is the target evaluation value actually deserved by the enterprise, the red line is the predicted value obtained by BPNN, and the blue line represents the error between the predicted value and the target value. From the overall trend, the fitting degree is high between the predicted value and the target value obtained by BPNN. The minimum error between them is 0.000436, the maximum is 0.01933, and the average is about 0.00873. Therefore, the deviation is small between the prediction result and the target value based on BPNN, the overall error is controlled within 0.02, and the prediction result is more accurate. This method has broad application prospects in evaluating the financing ability of HNTEs.

To sum up, the NLP-based innovation project document audit method proposed has higher recall rate and F statistical value and shorter information processing time than the manual processing method. This method can effectively improve the document management efficiency of enterprise innovation projects; The overall prediction error of the evaluation model based on AHP and BPNN is controlled within 0.02, which can accurately and objectively evaluate the financing ability of enterprises. The above methods can provide technical support for the optimization and improvement of social audit.

## 4. Conclusion

Based on the current situation that there is still a lack of effective methods to evaluate the financing ability of enterprises, the HNTEs are taken as the research objects, and the correlation between social auditing and enterprise technological innovation is investigated. The average accuracy rate of the proposed NLP-based innovation project document audit method is 91.36%, the average recall rate is 96.34%, and the average F statistical value is 95.34%. Among them, the recall rate and F statistical value are about 2.3% and 1.4% higher than manual processing, respectively. The processing time of a single document based on NLP is only 87.5 s. The processing time is nearly 50 times lower than that of manual processing, which greatly improves the processing efficiency of document information. The error of the BPNN model predicting the enterprise financing ability is controlled within 0.02, which can provide more accurate prediction results. It innovatively combines NLP technology with BPNN and applies it in the field of social auditing. In previous studies, the combination of NLP technology and BPNN has been widely used in the economic field, mostly at the theoretical level. There are few studies on the combination of the two in social auditing. However, this study combines the data of the Shenzhen Stock Exchange to analyze practical problems, which provides a reference for the application of NLP technology and BPNN in practical fields, and provides a path for the intelligent development of enterprise financing innovation. Due to the influence of many factors, the research only concentrates on the two levels of technological innovation investment and technological innovation management. The selected research samples are few, the indicators are less representative, there are only 2–3 second-level indexes, the coverage is narrow, and the combination of BPNN and NLP technology is not deep enough. In the later stage, it is necessary to expand the research sample, include more indicators for further research, refer to more previous literature, deepen the combination of NLP technology and BPNN, and provide significant technical support for promoting technological innovation and development of enterprises and optimizing social auditing. After further optimization, this research will be expected to be put into the intelligent development and construction of enterprises in the financial field.

## Figures and Tables

**Figure 1:** The structure of BPNN.

**Figure 2:** Audit content composition of total factor technological innovation of HNTEs (The blue parts are the two main modules studied).

**Figure 3:** Comparison between manual processing and NLP processing.

**Figure 4:** The evaluation of enterprise financing ability under different indexes: (a) based on the first-level index; (b) based on the second-level index.

**Figure 5:** Comprehensive evaluation results based on BPNN.

**Table 1:** The composition of financing capability index system based on enterprise innovation investment.

First-level index	Second-level index
Innovation (*I*)	*I*1: Composition of R & D personnel
	*I*2: Number of invention patents

Profit (*P*)	*P*1: Sales profit ratio
	*P*2: Return on equity

Management (*M*)	*M*1: Turnover of current assets
	*M*2: Total asset turnover
	*M*3: Management shareholding ratio

Growth (*G*)	*G*1: Operating income
	*G*2: Net profit growth
	*G*3: Total assets growth

Ensure (*E*)	*E*1: Current ratio
	*E*2: Proportion of intangible assets
	*E*3: Rate of capital accumulation

**Table 2:** Key terms of innovation project document contract.

Key clause number	Key clause name	Key clause number	Key clause name
*a*	Product name	*h*	Valuation base date
*b*	Master slave relationship of product structure	*i*	Minimum amount of individual initial subscription
*c*	Product operation form	*j*	Processing form of subscription interest
*d*	Risk return characteristics	*k*	First differential
*e*	Investment strategy	*l*	Pursue differential
*f*	Duration	*m*	Contractual securities broker
*g*	Difference of subscription amount	*n*	Redemption fee

**Table 3:** Expert judgment matrix based on the first-level index of financing capacity of HNTEs.

—	*I*	*P*	*M*	*G*	*E*
*I*	1	1/6	1/5	1/3	1/8
*P*	6	1	2	3	2
*M*	5	1/2	1	3	1/3
*G*	3	1/3	1/2	1	1/3
*E*	8	1/2	3	3	1

**Table 4:** Expert judgment matrix based on the second-level index of financing capacity of HNTEs.

—	*I*1	*I*2				—	*P*1				*P*2	
*I*1	1	1/5				*P*1	1				1/5	
*I*2	5	1				*P*2	5				1	
—												
—	*M*1	*M*2		*M*3		—		*G*1		*G*2		*G*3
*M*1	1	1/2		3		*G*1		1		1/3		4
*M*2	2	1		3		*G*2		3		1		9
*M*3	1/3	1/3		1		*G*3		1/4		1/9		1
—												
—			*E*1		*E*2				*E*3			
*E*1			1		2				1/4			
*E*2			1/2		1				1/3			
*E*3			4		3				1			

**Table 5:** Weight distribution results based on the first and second-level indexes.

First-level indexes	Weight	Second-level indexes	Weight	Comprehensive weight
*I*	0.039	*I*1	0.107	0.005
		*I*2	0.634	0.025

*P*	0.363	*P*1	0.083	0.031
		*P*2	0.336	0.122

*M*	0.188	*M*1	0.198	0.038
		*M*2	0.257	0.049
		*M*3	0.093	0.018

*G*	0.097	*G*1	0.252	0.026
		*G*2	0.681	0.068
		*G*3	0.068	0.008

*E*	0.316	*E*1	0.105	0.034
		*E*2	0.098	0.032
		*E*3	0.283	0.088

**Table 6:** Comprehensive rating results of companies studied.

No. of company	Rating results	No. of company	Rating results
1	0.522	11	0.267
2	0.446	12	0.258
3	0.362	13	0.253
4	0.348	14	0.252
5	0.332	15	0.228
6	0.327	16	0.215
7	0.324	17	0.187
8	0.319	18	0.151
9	0.295	19	0.150
10	0.284	20	0.092

## Data Availability

The data used to support the findings of this study are included within the article.
